The article "Antioxidant and Immunomodulatory Activities of Essential Oil Isolated from Anti-Upper Respiratory Tract Infection Formulation and Their Chemical Analysis" was retracted in 2023. Reasons: signs of a paper mill; compromised peer review; unreliable results or conclusions.

# Antioxidant and Immunomodulatory Activities of Essential Oil Isolated from Anti-Upper Respiratory Tract Infection Formulation and Their Chemical Analysis

**DOI:** 10.1155/2022/7297499

**Published:** 2022-07-31

**Authors:** Heming Fan, Lin Zhang, Yue Li, Cheang Soo Khoo, Donghe Han, Qingquan Liu, Ping Li, Xian Zhang

**Affiliations:** ^1^Beijing Hospital of Traditional Chinese Medicine, Capital Medical University, Beijing 100010, China; ^2^Beijing Institute of Chinese Medicine, Beijing 100010, China; ^3^Department of Instrument Management & Analysis, Beijing Institute for Drug Control, Beijing 102206, China; ^4^Wentworth Institute, 302-306 Elizabeth Street, Surry Hills, NSW 2010, Australia; ^5^Beijing Key Laboratory of Clinic and Basic Traditional Chinese Medicine on Psoriasis, Beijing 100010, China; ^6^Department of Instrument Management & Analysis, Beijing Port Drug Inspection Institute of the People's Republic of China, Beijing 102206, China; ^7^Beijing Institute for Drug Control, Beijing 102206, China; ^8^Beijing Center for Vaccine Control, Beijing 102206, China

## Abstract

This study evaluates the in vitro antioxidant and immunomodulation activities of essential oils isolated from an anti-upper respiratory tract infection (URTI) formulation with a view to their therapeutic potential. The chemical components of the essential oil were analysed by gas chromatography-mass spectrometry (GC-MS). The antioxidative activity of the oils was investigated with regard to their ability to scavenge DPPH^●^, ABTS^●+^, and hydroxyl free radical (•OH). Their immunostimulatory activities were determined using murine macrophage cells. The main components of the oil with pharmacological and biological activities include 1,8-eucalyptol (42.9%), patchouli alcohol (19.9%), trans-erinolide (9.2%), and guaiacol (5%). The oils displayed high DPPH, ABTS, and hydroxyl radical scavenging activities and anti-inflammatory activities by reducing tumour necrosis factor-*α* (TNF-*α*) and interleukin-6 (IL-6) production. The results indicate that essential oils have the potential to be used in products for anti-URTI treatment.

## 1. Introduction

Infection refers to the invasion of bacteria, viruses, fungi, parasites, and other pathogens into the human body and their growth and reproduction in the body, resulting in compromising the body's normal function, metabolism, and tissue structure, resulting in local tissue damage and systemic inflammatory response [1—7]. The outbreak of epidemics causes huge losses to human society, but there are often few drugs for their symptomatic treatment. So far, the clinical drugs used for the treatment of upper respiratory tract infection (URTI) are mainly Western medicines. Complementary or herbal medicines are more assessable and affordable to people in developing countries, so it is important to find complementary or alternative means of protection and treatment of URTI [3].

The article "Antioxidant and Immunomodulatory Activities of Essential Oil Isolated from Anti-Upper Respiratory Tract Infection Formulation and Their Chemical Analysis" was retracted in 2023. Reasons: signs of a paper mill; compromised peer review; unreliable results or conclusions.

Herbal essential oils, also known as volatile oils, are highly concentrated extracts of plants containing balsam glands, and essential oils from traditional Chinese medicine have unique medicinal properties [2, 8, 9]. These oils are mild and have a wide range of uses, with few side effects. They have reported functions of preventing infectious diseases, have antibacterial, anti-inflammatory, antioxidant, and antiseptic properties, reducing depression, and promoting cell metabolism and cell regeneration [6]. The combination of aromatherapy with other medical treatments is sometimes used in traditional Chinese medicine. This study is based on anti-URTI prescription developed by the Beijing Hospital of Traditional Chinese Medicine (BHTCM) affiliated to Capital Medical University. This prescription is mainly used in our hospital for acute tonsillitis and pharyngeal conjunctivitis, and the observed effect is quite good. The essential oil components in the formulation were extracted and modern analytical techniques were used to analyse the main chemical components. An in vitro investigation into its antioxidant and immune-enhancing activities was also conducted to support further characterisation and development of the formulation.

## 2. Materials and Methods

### 2.1. Materials

The BHTCM formula was provided by Dr Liu Qingquan, Director of Beijing Hospital of Traditional Chinese Medicine, China, and consists of herbs which mainly include *Artemisia argyi*, Agastache rugosus, *Angelica dahurica*, and Amomum cardamon.

### 2.2. Chemicals

The DPPH^●^, ABTS^●+^, 1,10-phenanthroline, H_2_O_2_, dimethyl sulfoxide (DMSO), 95% ethanol, ascorbic acid, 0.4% trypan blue, and lipopolysaccharide (LPS) were purchased from Sigma (Australia) and Lomb Scientific Pty Ltd. (Australia). The foetal bovine serum (FBS, Gibco, Australia), CCK-8 kits (Beyotime Institute of Biotechnology, China), antibiotics, and Dulbecco's modified Eagle's medium (DMEM) with gluMax were purchased from BD Bioscience. The other reagentswere tris-HCl (AMRESCO, USA), 2-hydroxy-1-ethanethiol (Sigma Aldrich, USA), sodium dodecyl sulfate (SDS, AMRESCO, USA), anti-IL-6 (CST, USA), anti-TNF-*α* (ABCAM, USA), anti-GAPDH (CST, USA), and albumin bovine V (AMRESCO, USA). The TNF-*α* and IL-6 (mouse), ELISA standards and antibodies were purchased from BD Bioscience (USA).

### 2.3. Essential Oil Extraction from BHTCM Formulation

500 g of the dry herbal mixture was powdered and placed into a 5 L round-bottomed flask, and 2 L purified water added, and the mixture was allowed to soak for 30 min. The flask was connected to a volatile oil extractor and the essential oils were extracted for 10 h by steam distillation according to the methodology described in Chinese Pharmacopoeia [10, 11]. Extraction is complete when the amount of volatile oil in the measuring device no longer increases. The distilled water-oil mixture was collected in a separatory funnel and kept at room temperature for 1 h until the oil and water layers were separated. The oil was collected in a brown glass bottle and anhydrous sodium sulfate added for drying and then stored in a 4°C refrigerator for further study. The extraction efficiency was calculated by

(1) $$\begin{array}{c} \text{Extraction efficiency}\left(\%\right)=\frac{V}{m}\times 100\%, \end{array}$$

where *V* is the volume (mL) of the oil extract and *m* is the dry weight (*g*) of the herbal mixture.

The article "Antioxidant and Immunomodulatory Activities of Essential Oil Isolated from Anti-Upper Respiratory Tract Infection Formulation and Their Chemical Analysis" was retracted in 2023. Reasons: signs of a paper mill; compromised peer review; unreliable results or conclusions.

The density of essential oil was measured using the method described in the Chinese Pharmacopoeia (2015) [11]. Five mL of distilled water was added to the cleaned pycnometer and the weight of water (M_water_) was recorded. Care was taken to ensure that there was no air bubble inside the pycnometer while weighing. The water was removed and the pycnometer dried. The same volume of oil was added to the pycnometer and weighed (M_oil_). Finally, specific gravity or relative density was calculated using the following equation:

(2) $$\begin{array}{c} \text{Density}=\frac{M_{\text{oil}}}{\;M_{\text{water}}}. \end{array}$$

### 2.4. Major Chemical Components of the Essential Oil from BHTCM Formulation

GC-MS analysis of the extracted oil was performed with some modifications to the method of Chen [12]. A TSQ Quantum XLS Thermogongsi GC-MS with HP-5MS capillary column (Agilent Technologies HP5-MS 30 m × 0.25 mm × 0.25 *µ*m film thickness) was used. The initial oven temperature was 50°C maintained for 4 min, increased to 120°C at the rate of 5°C/min and maintained for 1 min before being raised to 180 °C at the rate of 1°C/min, and finally to 280°C at the rate of 10°C/min. The injector temperature was 280°C and injection volume 0.2 *μ*L with a 1:10 split ratio. The carrier gas was helium at a flow rate of 1 mL/min. The oil sample was diluted 1:100 in anhydrous ethanol. The MS source temperature was 260°C, MS quadrupole temperature 150°C, ionization energy 70 eV, ionization current 50 *μ*A, and scan range 30–500 *m/z*. Identification of essential oil compounds was performed by comparing peaks from the total ion chromatogram with the commercial mass spectra libraries (NIST11). Relative amounts of individual components were calculated based on the peak areas.

The article "Antioxidant and Immunomodulatory Activities of Essential Oil Isolated from Anti-Upper Respiratory Tract Infection Formulation and Their Chemical Analysis" was retracted in 2023. Reasons: signs of a paper mill; compromised peer review; unreliable results or conclusions.

### 2.5. Antioxidant Activities Measurement

The DPPH^●^ scavenging activity test was determined by the Blois method [13]. 62.5 *μ*mol/L DPPH solution was prepared using 60% ethanol and stored at 4°C in the dark for future use. Absolute ethanol was used to prepare oils with different concentrations (0–1000 *μ*g/mL). Ascorbic acid (Vc) at a concentration range of 0-1 mg/mL was the positive control. 1.0 mL of sample mixed with 2 mL DPPH solution. After reacting at room temperature for 30 min in the dark, the absorbance at 517 nm was determined. Each sample was measured 3 times in parallel, and the average value was obtained [13–16].

Free radical scavenging activities of oil sample were evaluated using the following equation:

(3) $$\begin{array}{c} {\text{DPPH}}^{•}\text{scavenging activity}\left(\%\right)=\frac{{\text{OD}}_{\text{control}}-{\text{OD}}_{\text{sample}}}{{\text{OD}}_{\text{control}}}\times 100\%, \end{array}$$

where OD of the control is the absorbance of DPPH solution without sample and OD of sample is the test sample (DPPH solution plus test sample or positive control).

The ABTS^●+^ scavenging ability of the oil was determined using a published method and is similar to that described in previous publications [14–16].

Free radical scavenging activity of oil sample was evaluated using the following equation:

(4) $$\begin{array}{c} {\text{ABTS}}^{•+}\text{scavenging activity}\left(\text{\%}\right)=\frac{{\text{OD}}_{\text{control}}-{\text{OD}}_{\text{Sample}}}{{\text{OD}}_{\text{control}}}\times 100\text{\%,} \end{array}$$

where OD of the control is the absorbance of ABTS solution without sample and OD of sample is the test sample (ABTS solution plus test sample or positive control).

The OH^●^ scavenging assay is a slightly modified method of de Avellar et al. [17]and is described in previous publications[16, 17]. The OH^•^ scavenging ability of the oil sample was determined using the following equation:

(5) $$\begin{array}{c} OH^{•}\text{scavenging activity}\left(\%\right)=\frac{{\text{OD}}_{\text{Sample}}-{\text{OD}}_{\text{neg\_control}}}{{\text{OD}}_{\text{blank}}-{\text{OD}}_{\text{neg\_control}}}\times 100\%, \end{array}$$

where the negative control is the reaction mixture without sample and ascorbic acid. The blank is the reaction mixture without sample, ascorbic acid, and H_2_O_2_.

### 2.6. Immunomodulatory Activities Assay

Mouse macrophage cell RAW 264.7 was cultured using a complete medium (DMEM high glucose medium supplemented with 10% (*v/v*) fetal bovine serum, 100* *U/mL penicillin, and 100* μ*g/mL streptavidin). The cells were cultured in an incubator at 37°C with 5% CO_2_ and passaged every 2 days. The RAW 264.7 cells in the logarithmic growth phase were adjusted to a cell density of 2 × 10^4^ cells/mL and seeded in 96-well plates at 100 *μ*L/well. After culturing for 18 h, the original medium was removed and 100* μ*L of new medium added to determine the production of IL-6 and TNF-*α* and the cytotoxicity test [18–21]. To 50 *μ*L of the sample (900 *μ*g/*μ*L), 5 *μ*L of DMSO was added and mixed well before adding 445 *μ*L of culture medium and vortexed for 1 min to prepare a stock solution of the test sample with a concentration of 90 *μ*g/*μ*L.

The article "Antioxidant and Immunomodulatory Activities of Essential Oil Isolated from Anti-Upper Respiratory Tract Infection Formulation and Their Chemical Analysis" was retracted in 2023. Reasons: signs of a paper mill; compromised peer review; unreliable results or conclusions.

#### 2.6.1. Determination of Cell Viability by CCK-8

The viability of macrophage cells (RAW 264.7) was measured using the CCK-8 assay following the method provided in the manufacturer's manual and published papers [22, 23]. The absorbance at 450 nm was measured and the fraction of live cells was determined using the following equation:

(6) $$\begin{array}{c} \text{Cell viability}\left(\%\right)=\frac{\text{OD of sample}}{\text{OD of pos control}}\times 100\%. \end{array}$$

The positive control was mouse macrophages treated by DMEM medium only (without LPS and sample).

#### 2.6.2. Inhibition of IL-6 Activity

The assay for inhibition of IL-6 activity was performed in mouse macrophages (RAW264.7) [20, 21]. Cells were plated at a density of 20,000 cells/well and incubated for 24 h for confluency. Oil samples with final concentrations of 9000, 2000, 500, 100, 50, and 20 ng/*μ*L were added to the cells. After 30 min incubation, the cells were induced with LPS (1 *μ*g/mL) for 24 h (LSP group). ELISA kit (TNF-*α*, BD Biosciences, San Jose, CA, USA) was used to measure the concentration of IL-6 following the method provided in the manufacturer's manual and as previously described [16, 18–21]. Triplicate measurements were conducted.

Standard TNF-*α* (mouse) was used to produce the calibration curve that gave the linear equation (*R*^2^ = 0.9959):

(7) $$\begin{array}{c} y=426.77x-24.731. \end{array}$$

The IL-6 production percentage inhibition was calculated using the following equation:

(8) $$\begin{array}{c} \text{IL}-6\text{ inhibition}\left(\%\right)=\left(1-\frac{{\text{OD}}_{\text{samples}}-{\text{OD}}_{\text{blank}}}{{\text{OD}}_{\text{LPS}}-{\text{OD}}_{\text{blank}}\;}\right)\;\times 100\%. \end{array}$$

#### 2.6.3. Inhibition of TNF-*α* Activity

The assay for inhibition of IL-6 activity was performed using mouse macrophages (RAW264.7). Cells were plated at a density of 20,000 cells/well and incubated for 24 h for confluency. Oil samples with a final concentration of 9000, 2000, 500, 100, 50, and 20 ng/*μ*L were added to the cells. After 30 min incubation, the cells were induced with LPS (1 *μ*g/mL) for 24 h (LSP group). ELISA kit (TNF-*α*, BD Biosciences, San Jose, CA, USA) was used to measure the concentration of TNF-*α* following the method provided in the manufacturer's manual and as previously described [16, 18–21]. Triplicate measurements were conducted.

The article "Antioxidant and Immunomodulatory Activities of Essential Oil Isolated from Anti-Upper Respiratory Tract Infection Formulation and Their Chemical Analysis" was retracted in 2023. Reasons: signs of a paper mill; compromised peer review; unreliable results or conclusions.

Standard TNF-*α* (mouse) was used to produce the calibration curve that gave the linear equation (*R*^2^ = 0.9936):

(9) $$\begin{array}{c} y=411.67x+17.327, \end{array}$$

which was used to determine the concentration of TNF-*α* produced by the oil extract-treated sample.

The IL-6 production percentage inhibition was calculated using the following equation:

(10) $$\begin{array}{c} \text{TNF}-\alpha \text{ inhibition}\left(\%\right)=\left(1-\frac{{\text{OD}}_{\text{samples}}-{\text{OD}}_{\text{blank}}}{{\text{OD}}_{\text{LPS}}-{\text{OD}}_{\text{blank}}\;}\right)\times 100\%.\; \end{array}$$

#### 2.6.4. Western blot Tests

To investigate the inhibitory effect of the essential oil sample on IL-6 and TNF-*α* production in LPS-stimulated RAW 264.7, the cells were pretreated with the oil (20, 50, and 100 ng/*μ*L) for 60 min at 37°C, followed by LPS (1 *µ*g/mL) treatment for 24 h. The cells were immediately pelleted at 4°C and lysed with 300 *µ*L of ice-cold lysis buffer (50 mM tris-HCl, pH 8.0, 150 mM NaCl, 1% Triton, 0.5% sodium deoxycholate, 0.1% sodium dodecylsulphate, and protease inhibitors) on ice for 30 min. Insoluble material was removed by centrifugation at 4 °C for 15 min at 12000 g. At the same time, it was compared with the cells without LPS treatment (only treated with 20, 50, and 100 ng/*μ*L oil sample) and those without the oil and LPS treatment (control group). The protein concentrations were determined using a Bio-Rad protein assay. The detailed information on the Western blotting method is provided in the manufacturer's manual used as previously described [24–25]. The results were analysed using Image J (National Institutes of Health, USA) and GraphPad Prism 9.0 (GraphPad InStat or Sigma Stat).

### 2.7. Statistical Analysis

Data are expressed as mean ± standard deviation (SD) values. The group mean was compared using a one-way analysis of variance (ANOVA) and Duncan's multiple range tests. The statistical difference was considered significant if *p* < 0.05. All statistical analyses were performed using OriginPro 8.5, Image J, GraphPad Prism 9.0, and Excel 2016.

## 3. Results and Discussion

### 3.1. Extraction Efficiency and Main Chemical Components of Essential Oils in the BHTCM Formulation

Using the equipment described in Section 3.3, the average extraction efficiency of the essential oil is 1.12% and the density is 0.9732 g/mL. The chemical composition of the essential oil extract from the BHTCM formulation was analysed by GC-MS, and the results are given in Table 1 and Figure 1.

The article "Antioxidant and Immunomodulatory Activities of Essential Oil Isolated from Anti-Upper Respiratory Tract Infection Formulation and Their Chemical Analysis" was retracted in 2023. Reasons: signs of a paper mill; compromised peer review; unreliable results or conclusions.

Using the GC-MS NIST11 mass spectral library and manual analysis with standard mass spectra, 12 main essential oil chemical components were identified, and their relative contents were calculated by the area normalization method. It is noted that the area normalization method assumes that the detector response is constant for all the essential oils of interest. Only clearly identified peaks were included in the calculation. Table 1 provides the active ingredients, and their relative percentages. These are 1,8-eucalyptol(42.9%), patchouli alcohol (19.9%), trans-citronolide (9.2%), *α*-bulinene (5.8%), *α*-guaiene (5%), *α*-terpineol (4.1%), *β*-patchoulene (3.1%), and (−)-*α*-pinene (2.9%).

### 3.2. Antioxidant Activities of the Essential Oil

The DPPH radical has a single electron, and its ethanolic solution is dark purple with strong absorption at 517 nm. The presence of antioxidants makes the colour of DPPH solution change from dark purple to light yellow, which indicates their ability to scavenge DPPH free radicals—the more obvious the fading, the stronger the antioxidant ability [15].

The ABTS radical has a strong absorption at 734 nm. The presence of antioxidants makes the colour of ABTS solution change from blue to colourless, indicating their ability to scavenge ABTS free radicals—the more obvious the fading, the stronger the antioxidant ability [15].

•OH is a highly oxidizing active oxygen free radical, which mainly undergoes a series of oxidative reactions and abstracts H-atoms through electron transfer, which accelerates the oxidation of proteins, lipids, and carbohydrates, causing peroxidative damage to organisms [17, 26]. The antioxidant activity of the test sample was measured by its ability to scavenge •OH. The absorbance of the sample at 536 nm is proportional to the antioxidant ability.

The free radical scavenging activities of the essential oil compared to that of the ascorbic acid standard are shown in Figure 2. The results are presented as a percentage of the scavenging activity of ascorbic acid which is taken as 100%. The results indicate that the oil has high DPPH^●^ and ABTS^●+^ free radical scavenging abilities (Figure 2(a) and Figure 2(b)). The essential oil at the maximum concentration was most active against DPPH^●^ at 52%. The activity against ABTS^●+^ radical was 59%. The EC50 value of the oil for DPPH free radical is about 995 *µ*g/mL, and the EC50 value for ABTS free radical is about 571 *µ*g/mL. The OH• scavenging ability is shown in Figure 2(c). The oil exhibited very high OH• radical scavenging activity (>70%) with an EC50 value of approximately 415 *µ*g/mL.

The article "Antioxidant and Immunomodulatory Activities of Essential Oil Isolated from Anti-Upper Respiratory Tract Infection Formulation and Their Chemical Analysis" was retracted in 2023. Reasons: signs of a paper mill; compromised peer review; unreliable results or conclusions.

According to literature reports [27–29], the antioxidant mechanism of essential oils is mainly related to its antioxidant components such as polyphenols, vitamins, alkaloids, saponins, polysaccharides, polypeptides, and terpenes. The mechanism mainly includes three aspects, namely, they directly scavenge free radicals, inhibit the generation of free radicals, and activate the antioxidant system. The results of this study indicate that the essential oil displayed good antioxidant activity, which is most likely related to the presence of a large amount of terpenoids and olefins, especially the olefins that contain -C=C- which can effectively capture free radicals [27–29]. However, the DPPH, ABTS, and hydroxyl radical scavenging activities of the essential oils were weaker than those of ascorbic acid.

### 3.3. Immunostimulation Activities Test

#### 3.3.1. CCK-8

Figure 3 shows the effect of the essential oil from the BHTCM formulation on the viability of mouse macrophage cells (RAW 264.7). The results show that the inhibitory concentration (IC50) value on cell activity was 394.5 ng/*μ*L, indicating that the concentration of the oil should be less than 394.5 ng/*μ*L for future studies.

#### 3.3.2. Anti-Inflammatory Activity

LPS can stimulate a variety of cells such as smooth muscle cells, macrophages, and hepatocytes and induce immune cells to generate various immune signals such as IL-6 and TNF-*α* [30]. The production of IL-6 and TNF-*α* can indicate inflammatory damage [18]. As shown in Figure 4, the production of IL-6 and TNF-*α* in the essential oil was significantly lower (*p* < 0.05) than that in the LPS treatment group. The overall production showed a downward trend. The results showed that when the oil was at the maximum safe concentration (100 ng/*μ*L), the production of IL-6 in the oil sample group compared with the LPS group decreased by 61% (Figure 4(b)), and the generation of TNF-*α* reduced by 57% (Figure 4(c). Treatment of RAW 264.7 cells with 20 and 100 ng/*µ*L of the oil for 24 h significantly reduced IL-6 and TNF-*α* protein expression (Figures 5(a) and 5(b)). These results indicated that the oil significantly alleviated the inflammatory state of LPS-induced RAW 264.7 cells at the tested concentrations in a dose-dependent manner.

The main components of the oil are 1,8-eucalyptol (42.9%) and patchouli alcohol (19.9%). According to literature reports [21, 28, 31], eucalyptol and patchouli alcohol intervene on inflammatory-related targets, including inhibition of cyclooxygenase (COX)-2, inducible nitric oxide synthase (iNOS), toll-like receptor (TLR), and nuclear factor-*κ*B (nuclear factor-*κ*B, NF-*κ*B) signalling pathway expression and activation, reduce the synthesis and release of inflammatory mediators, and regulate oxidative stress and immune response. Studies have also shown that eucalyptol can significantly reduce proinflammatory factors, such as nitric oxide (NO), tumour necrosis factor (TNF-*α*), interleukin (interleukin, IL)-1*β*, IL-6, and interferon (interferon, IFN)-*γ* [28]. The results of this study also showed that the oil containing 1,8-eucalyptol and patchouli alcohol has excellent anti-inflammatory abilities. Therefore, in the future, the essential oils from BHTCM may be further developed as potential anti-inflammatory functional products.

The article "Antioxidant and Immunomodulatory Activities of Essential Oil Isolated from Anti-Upper Respiratory Tract Infection Formulation and Their Chemical Analysis" was retracted in 2023. Reasons: signs of a paper mill; compromised peer review; unreliable results or conclusions.

## 4. Conclusion

Studies have shown that the main compounds of essential oils in the BHTCM formula are 1,8-eucalyptus and patchouli alcohol. When studying the in vitro antioxidant activity of the oil, it was found to have strong antioxidant activities, though less than ascorbic acid and contain olefins. The oil also had good in vitro anti-inflammatory ability, especially at a concentration of 394 ng/*μ*L. Its anti-inflammatory activity may be related to the main chemical components 1,8-eucalyptol and patchouli alcohol contained in the oil formula. The oil extract of the BHTCM formula is a promising candidate for further research and development as an anti-inflammatory and immune-enhancing product.

## Figures and Tables

**Figure 1:** Total ion chromatogram of the essential oil from BHTCM formulation.

**Figure 2:** Antioxidant activities of essential oil from BHTCM formulation. (a) DPPH free radical scavenging activity. (b) ABTS free radical scavenging activity. (c) Hydroxyl radical scavenging activity. All the results are compared with standard (ascorbic acid) in a line chart.

**Figure 3:** Effect of the essential oils on RAW 264.7 cells viability.

**Figure 4:** Effect of essential oil on IL-6 ((a)-(b)) and TNF-*α* production ((c)-(d)) in LPS-stimulated macrophages. Each value represents the mean ± SEM of three independent assays made in triplicate (^*∗*^*p* < 0.05 compared with LPS).

**Figure 5:** Relative expression levels of the IL-6 protein and (a) TNF-*α* protein in RAW 264.7 cells treated with essential oil (b). Each panel shows the densitometry of bands in the treated groups and control. Values are the mean ± SD in each group (*n* = 3). ^*∗*^*P* < 0.01, ^*∗∗*^*p* < 0.03, ^*∗∗∗*^*p* < 0.0005 compared to control (ANOVA followed by Dunnett's multiple comparison test).

**Table 1:** Major chemical compositions of the essential oil from BHTCM formulation^*∗*^.

BHTCM formulation					
Peak no.	Retention time (min)	Compounds	Molecular formula	Constitution of total essential oil (%)	Similarity (%)
1	9.31	(−)-*α*-Pinene	C_10_H_16_	2.9	91.1
2	11.12	1, 8-Eucalyptol	C_10_H_18_O	42.9	92.0
3	15.65	(−)-4-Terpineol	C_10_H_18_O	2.6	86.5
4	16.05	*α*-Terpineol	C_10_H_18_O	4.1	82.3
5	22.27	*β*-Patchoulene	C_15_H_24_	3.2	84.2
6	23.92	*β*-Caryophyllene	C_15_H_24_	1.9	82.0
7	24.58	(−)-*γ*-Elemene	C_15_H_24_	2.0	84.0
8	24.85	*α*-Guaiene	C_15_H_24_	5.1	83.6
9	26.75	Dodecanol	C_12_H_16_O	0.33	83.7
10	28.35	*α*-Bulinene	C_15_H_24_	5.9	80.3
11	37.81	Patchouli alcohol	C_15_H_26_O	19.9	90.6
12	43.99	*trans*-Citronolide	C_12_H_14_O_2_	9.2	92.9

^*∗*^Very small quantities or uncertain components in essential oil are not presented in the table.

The article "Antioxidant and Immunomodulatory Activities of Essential Oil Isolated from Anti-Upper Respiratory Tract Infection Formulation and Their Chemical Analysis" was retracted in 2023. Reasons: signs of a paper mill; compromised peer review; unreliable results or conclusions.

## Data Availability

The data used to support this study are available from the corresponding author upon request.
